The article "Comprehensive and Integrated Analysis Identifies ZEB1 as a Key Novel Gene in Oral Squamous Cell Carcinoma" was retracted in 2023. Reasons: signs of a paper mill; suspected computer-generated content; unreliable results or conclusions; concerns about the data.

# Comprehensive and Integrated Analysis Identifies ZEB1 as a Key Novel Gene in Oral Squamous Cell Carcinoma

**DOI:** 10.1155/2022/4486104

**Published:** 2022-08-09

**Authors:** Jie Ma, Yu Yao, De-tao Tao, Jia-yi Yin, Liang Chen, Yong Cui, Ying Wang, Cong-lin Hu, Ming-xing Tian, Qiong Wang

**Affiliations:** ^1^Department of Stomatology, The First Affiliated Hospital of Wannan Medical College, Wuhu, Anhui 241001, China; ^2^Wannan Medical College, Wuhu, Anhui 241000, China

## Abstract

Oral squamous cell carcinoma (OSCC) is the most common head and neck cancer with a poor prognosis. Therefore, it is crucial to explore molecular prognostic biomarkers for OSCC. ZEB1 (also known as *δ*EF1) is a member of the zinc finger E-box binding protein family of transcription factors involved in various biological processes, including tumorigenesis, progression, and metastasis. Recent evidence suggests that ZEB1 has a role in the tumorigenicity of oral epithelial cells, although its mode of action needs to be investigated further. To better understand the relationship between ZEB1 and OSCC, we transfected the ZEB1-overexpressing oral squamous cell lines SCC9 and SCC25 with lentivirus and then extracted RNA from the cells for gene expression analysis. Furthermore, the GSE30784 dataset was downloaded from the Gene Expression Omnibus (GEO) database to identify potential biomarkers of OSCC and to assess the potential mechanisms. The criteria for identification of their DEGs were |logFC| > 1 and *P* < 0.05. Gene Ontology (GO) and Kyoto Encyclopaedia of Genes and Genomes (KEGG) analyses were also carried out. Integrating the data from the PPI network and survival analysis identified that ZEB1 might be an independent prognostic biomarker in OSCC. In conclusion, integrated bioinformatics and microarray analysis identified the critical gene ZEB1 linked to the overall survival (OS) of patients with OSCC. ZEB1 could be applied as a prognostic biomarker to forecast the survival of patients with OSCC and might indicate innovative therapeutic indicators for OSCC.

## 1. Introduction

Oral squamous cell carcinoma (OSCC) is a common type of head and neck cancer, accounting for approximately 90% of all oral malignancies [1]. Despite improvements in surgical techniques, chemoradiotherapy, and immunotherapy, the five-year survival rate for patients with OSCC is still only approximately 50% over the past decade, and 25%–50% of the patients might be afflicted by distant metastases after surgery [2]. OSCC is a rapidly progressive disease with a high incidence and poor diagnosis, and numerous researchers have carried out comprehensive studies on the incidence and prospective remedial targets for OSCC [3, 4]. It is critical to find tumor-specific biomarkers and probable molecular mechanisms for OSCC, which might contribute to improving risk assessment, therapy regimens, novel diagnostics, and treatments for the disease.

The article "Comprehensive and Integrated Analysis Identifies ZEB1 as a Key Novel Gene in Oral Squamous Cell Carcinoma" was retracted in 2023. Reasons: signs of a paper mill; suspected computer-generated content; unreliable results or conclusions; concerns about the data.

Chromatin immunoprecipitation (ChIP) combined with microarray technology is an efficient method that has been widely used for gene expression profiling [5]. In recent years, many studies have used microarray analysis to explore the differentially expressed genes (DEGs) and functionally enriched pathways associated with the development and progression of OSCC that might serve as underlying biomarkers for diagnosing or treating OSCC [6, 7]. Kinouchi et al. established a high-throughput system for the identification of OSCC etiology and obtained nine molecular indicators to distinguish salivary SCC [8]. Through microarray analysis, Ren et al. exposed the controlling mechanisms of miRNAs and matrix metalloproteinases (MMPs) in OSCC [9]. Fang et al. characterized the differential expression of lncRNAs in OSCC tissues and normal tissues by RNA-Seq [10]. Additionally, Ganesan et al., based on The Cancer Genome Atlas (TCGA) database data, identified dysfunctional lncRNAs in OSCC that were correlated with smoking history using microarray analysis [11].

ZEB1 (also known as *δ*EF1, AREB6, ZFHEP, ZFHX1A, BZP, NIL-2-A, and DeltaEF1) is a member of the zinc finger E-box binding protein family transcription factors that has critical functions in the metastasis of some epithelial cancers, such as pancreatic cancer [12], prostate cancer [13], epithelial ovarian cancer [14], and nonsmall cell lung cancers [15]. Recent evidence supports the role of ZEB1 in the tumorigenicity of oral epithelial cells, but its potential mechanism of action needs further investigation.

In the current study, we evaluated datasets retrieved from TCGA and GEO and performed microarray analysis to explore the association between ZEB1 expression and the clinical and pathological features of OSCC. Furthermore, we found that ZEB1 affects the clinical characteristics of patients with OSCC.

## 2. Materials and Methods

### 2.1. Data Sources

Data were obtained from The Cancer Genome Atlas (TCGA), Gene Expression Omnibus (GEO), and Genotype-Tissue Expression (GTEx), containing clinical and gene expression matrix data. A total of 214 OSCC samples were obtained from the TCGA database, 167 tumor tissues were obtained from the GSE30784 dataset, and 33 cancer samples were obtained by integrating the TCGA and GTEx datasets.

### 2.2. Differential Analysis

The data were normalized using *R* software (version 2.6.0). The genes with an |FC| > 2.0 and an adjusted *P* < 0.05 between OSCC and normal were specified as differentially expressed genes (DEGs).

The article "Comprehensive and Integrated Analysis Identifies ZEB1 as a Key Novel Gene in Oral Squamous Cell Carcinoma" was retracted in 2023. Reasons: signs of a paper mill; suspected computer-generated content; unreliable results or conclusions; concerns about the data.

### 2.3. Analysis of ZEB1 Expression and Survival in Each Tumor

The Kruskal-Wallis test was used to analyze the differences between tumor tissues and normal tissues. *P* < 0.05 was considered statistically significant.

### 2.4. Functional and Pathway Enrichment Analysis

DEG functional and pathway enrichment and annotation were performed using DAVID (https://david.ncifcrf.gov/). Enrichment analyses, such as Gene Ontology (GO) and Kyoto Encyclopaedia of Genes and Genomes (KEGG) pathways, were carried out using the cluster Profiler package. The statistical significance was set at *P* < 0.05.

### 2.5. Protein-Protein Interaction Network Construction

The PPI among DEGs was carried out using the Search Tool for the Retrieval of Interacting Genes and proteins (STRING) database (ver. 10.0, http://www.string-db.org/). The network visualization software Cytoscape (http://www.cytoscape.org/) was applied to create the PPI interaction network.

The top 100 genes were chosen as the hub genes through the CytoHubba plugin of Cytoscape.

### 2.6. Survival Analysis and Cox Regression Analysis

We assessed the impact of the expression levels of ZEB1 on the OS of patients with OSCC. Patients were divided into low- and high-expression groups according to the median ZEB1 expression. The accuracy of the Cox mark was evaluated by receiver operating characteristic (ROC) analysis using the *R* package. The prognostic values of the low- and high-expression groups were assessed using Kaplan–Meier (KM) curves in the survival *R* package. *P* < 0.05 was considered the cut-off criterion.

### 2.7. Illumina Microarrays Analysis

SCC9 and SCC25 cells were transfected with lentivirus-mediated ZEB1 overexpression or the negative control (Shanghai Genechem) for 14 hours. Five hundred nanograms of RNA were amplified and labeled using the Illumina® TotalPrep™-96 RNA Amplification Kit (Life Technologies). BeadChips were scanned in an Illumina Scanner.

### 2.8. Analysis of Association with Tumor Immunity

TIMER was applied to validate the association between ZEB1 and tumor-infiltrating immune cells. The Pearson correlation coefficient was employed to estimate the extent of correlation between tumor immunity and ZEB1. The ggplot2 and reshape2 in the *R* package were used to plot and visualize the results.

## 3. Results

### 3.1. Identification of DEGs in OSCC Based on the GEO Database

The mRNA microarray dataset GSE30784 of the GEO database was used to evaluate significant genes and pathways involved in OSCC. THE DEGs were identified using the limma package, |logFC| > 1 and *P* < 0.05. A total of 530 DEGs were identified in the GSE30784 dataset. A volcano plot was generated in the GSE30784 dataset showing the distribution of these DEGs (Figure 1(a)). The clustered heat map exhibited the different displays of OSCC and normal samples (Figure 1(b)). ZEB1 was identified as a differentially expressed gene involved in OSCC.

The article "Comprehensive and Integrated Analysis Identifies ZEB1 as a Key Novel Gene in Oral Squamous Cell Carcinoma" was retracted in 2023. Reasons: signs of a paper mill; suspected computer-generated content; unreliable results or conclusions; concerns about the data.

### 3.2. Functional Enrichment Analysis Based on GEO Database

To explore the molecular mechanisms associated with OSCC, we performed a functional enrichment analysis on these DEGs. These DEGs were interred into the online tool DAVID for GO enrichment analysis. The results showed that the upregulated DEGs (Figure 2(a)) were significantly enriched in biological processes (BP) “G-protein-coupled receptor signaling pathway,” “proteolysis,” “cell surface receptor signaling pathway,” and “cellular protein metabolic processes,” “regulation of ion transport across membranes,” and in the cellular components “integral components of membranes,” “plasma membrane,” “extracellular matrix” and molecular functions “G-protein-coupled receptor activity,” “metalloendopeptidase activity,” and “ion channel binding.” Moreover, downregulated DEGs (Figure 2(b)) were mainly enriched in biological processes (BP) “transmembrane transport,” “chemical synaptic transmission,” “sodium ion transport,” and cellular components “glutamatergic synapses,” “receptor complexes,” “basolateral plasma membrane,” and molecular functions “signaling receptor activity,” and “cation channel activity.” Furthermore, in KEGG enrichment analysis, vascular smooth muscle contraction, protein digestion and absorption, and cGMP-PKG signaling pathways were significantly enriched by these DEGs (Figure 2(c)).

### 3.3. PPI Network Construction and Subnetwork Module Analysis Based on the GEO Database

The PPI network of these DEGs was constructed by STRING and visualized through Cytoscape. The results showed that the PPI enclosed 108 nodes and 470 PPI pairs (Figure 3). Based on the data from STRING, 100 genes were selected as hub genes and exposed to a strong connection with other nodes. Importantly, we focused on the ZEB1 gene as a key pivotal gene in oral squamous cell carcinoma.

### 3.4. ZEB1 Was Expressed in Most Tumor Tissues

As shown in Figure 4, ZEB1 was markedly expressed in all 33 tumor cell lines. Integration of data in TCGA and GTEx revealed that ZEB1 expression was upregulated in 19 tumors, including DLBC, LGG, PAAD, THYM, and GBM, and was downregulated in 14 tumors, including BLCA, CESC, and COAD, among 33 tumor types.

### 3.5. Evaluation of ZEB1 in Oral Cancer-Based TCGA Database

In this study, we used samples from the TCGA database to investigate the mRNA expression levels of ZEB1 in oral tissues and its clinical significance.  Table 1 showed the correlation of ZEB1 expression with clinicopathological features in the GSE30784 dataset. Figure A is a univariate analysis of the prognostic value of ZEB1 expression in oral squamous cell carcinoma. The mRNA levels of ZEB1 were higher in OSCC tissues than in adjacent normal tissues (*P* < 0.05, Figure 5(b)). The mRNA expression of ZEB1 was higher in advanced-stage patients (III-IV) than in early-stage patients (I-II) (Figure 5(c), *P* < 0.01). The survival analysis of the ZEB1 gene was performed using univariate Cox analysis. The impact of ZEB1 on the 5-year survival rate in OSCC patients was investigated by allocating patients into two groups with higher or lower ZEB1 gene expression (median was considered as the cut-off). The results showed the significance of ZEB1 as a prognostic factor in OSCC patients. We found that patients with higher ZEB1 gene expression had a poorer 5-year survival rate than patients with lower ZEB1 gene expression and the difference was statistically significant (Figure 5(d), *P* < 0.05). ROC showed that the expression of ZEB1 mRNA in OSCC was 0.572 (95% CI: 0.474–0.670) (Figure 5(e)). In order to investigate the application of ZEB1 in cancer prognosis, we built a nomogram for predicting the overall survival of OSCC patients in the TCGA cohort. The cancer stage and ZEB1 were included as prognostic factors in the nomogram (Figure 5(f)). These results suggest that ZEB1 is overexpressed in OSCC tissues and that ZEB1 expression correlates with the clinical characteristics of the tumor.

The article "Comprehensive and Integrated Analysis Identifies ZEB1 as a Key Novel Gene in Oral Squamous Cell Carcinoma" was retracted in 2023. Reasons: signs of a paper mill; suspected computer-generated content; unreliable results or conclusions; concerns about the data.

### 3.6. Microarray Analysis and Screening of DEGs in OSCC

To further evaluate the effect of ZEB1 on OSCC gene expression profiles, we transfected oral squamous cell lines SCC9 and SCC25 with lentivirus-mediated ZEB1 overexpression and evaluated the gene expression profiles in transfected cells using Illumina microarray analysis. Volcano plots were applied to show the DEGs of SCC9 and SCC25 cell lines (Figures 6(a) and 6(b)). The heat map showed 1320 DEGs for SCC9 and 1456 DEGs for the SCC25 cell line (Figures 6(c) and 6(d)). A total of 74 upregulated genes and 72 downregulated genes were identified by the combined analysis, as shown in the Venn diagram (Figures 6(e) and 6(f) and Table 2).

### 3.7. Molecular Mechanisms of OSCC

The pathways of cell lines SCC9 and SCC25 were obtained by GO and KEGG enrichment analysis. The results of the Go pathways for the SCC9 cell line were exhibited in Figure 7(a), including the biological processes (BP) “cellular component organization or biogenesis,” “metabolic process,” “metabolic process,” “immune system process,” “biological regulation,” and cellular component (CC) “membrane-enclosed lumen,” “organelle part,” “extracellular region part,” “membrane part,” and molecular functions (MF) “nucleic acid binding transcription factor activity,” “catalytic activity,” “structural molecule activity.” Similarly, the results of the Go pathway in SCC25 cells are shown in Figure 7(b). In addition, the results of the KEGG pathway for SCC9 and sSCC25 cell lines are shown in Figures 7(c) and 7(d).

The article "Comprehensive and Integrated Analysis Identifies ZEB1 as a Key Novel Gene in Oral Squamous Cell Carcinoma" was retracted in 2023. Reasons: signs of a paper mill; suspected computer-generated content; unreliable results or conclusions; concerns about the data.

### 3.8. Correlation of ZEB1 with Tumor-Infiltrating Immune Cells

TIMER database was employed to examine the association between the prognosis of ZEB1 and the infiltration of immune cells in OSCC (Figure 8). The association of B cells with the risk score was 0.295, and the association of CD8+ *T* cells with the risk score was 0.235. The association of CD4+ *T* cells with the risk score was 0.511. The correlation of purity with the risk score was −0.718. The correlation of macrophage and neutrophil with the risk were 0.556 and 0.299, respectively. These findings indicated that the prognosis of ZEB1 was notably associated with tumor-infiltrating immune cells.

## 4. Discussion

Oral squamous cell carcinoma (OSCC) is the leading cause of cancer-related deaths worldwide [16]. Extensive lymph node metastasis in OSCC is associated with low survival rates. Despite advances in the diagnosis and treatment of OSCC in recent decades, its five-year survival rate remains low [18]. With the development of bioinformatics, the understanding of OSCC has gradually broadened and deepened [19, 20]. Chai et al. performed a genome-wide CRISPR-Cas9 screen of OSCC cells and identified YAP1 and WWTR1 as key genes [21]. Amiri-Dashatan et al. explored the gene interactions and pathways in the development of OSCC, revealing the important genes and microRNAs interactions [22]. Puttipanyalears et al. identified DNA methylation biomarkers of OSCC by bioinformatics analysis [23].

The current study aimed to determine essential genes and pathways involved in OSCC using integrated bioinformatics analysis and microarray analysis. The GSE58812 dataset, which contains OSCC, was chosen for the current study. To assess the DEGs, the mRNA profile of GSE30784 was downloaded from the GEO database, and 530 DEGs were identified. Moreover, GO and KEGG pathway enrichment analyses were performed to functionally annotate genes and showed that the DEGs were principally enriched in the G-protein-coupled receptor signaing pathway, proteolysis, the cell surface receptor signaing pathway, and the cellular protein metabolic process. A PPI network was generated to show the interactions of the DEGs, such as ZEB1, SCN7A, PAPPA, KRT4, GPR123, and FA2H. ZEB1, a crucial member of the ZEB family of transcription factors, has been suggested to be a critical inducer of the epithelial-mesenchymal transition (EMT) [12]. ZEB1 can regulate target gene transcription by distinctive function types. In recent years, a growing body of evidence has shown that targeting ZEB1 could decrease the tumor cell invasion and proliferation [25]. Remarkably, it has been shown recently that ZEB1 could serve as a prognostic marker for patients with breast cancers [26]. EMT is a necessary process of cell remodeling characterized by loss of epithelial phenotype and increased mesenchymal phenotype [27]. ZEB1 is abnormally expressed in various human cancers and is best known for activating EMT in cancer cells to facilitate tumor development [28]. In recent years, a growing body of evidence has shown that EMT is involved in the pathogenesis of OSCC [29, 30]. As a crucial transcription factor of EMT regulation, we speculated that ZEB1 might play a critical role in the pathogenesis of OSCC. Evidence has indicated that ZEB1 expression was more potent in OSCC cells [31], but its potential mechanism of function demands further investigation. This study found that ZEB1 was noticeably expressed in all 33 tumor cell lines. Integration of data exposed upregulation of ZEB1 in 19 tumors, including DLBC, LGG, PAAD, THYM, and GBM, and downregulated in 14 tumors, including BLCA, CESC, and COAD, among 33 tumor types. Moreover, we found that patients with higher ZEB1 gene expression had a lower 5-year survival rate than patients with lower ZEB1 gene expression. These findings implied that ZEB1 might be considered a diagnostic and prognostic indicator in OSCC and could be applied for targeting the treatment of OSCC.

The article "Comprehensive and Integrated Analysis Identifies ZEB1 as a Key Novel Gene in Oral Squamous Cell Carcinoma" was retracted in 2023. Reasons: signs of a paper mill; suspected computer-generated content; unreliable results or conclusions; concerns about the data.

To further evaluate the effect of ZEB1 on the gene expression profile of OSCC, the oral squamous cell lines SCC9 and SCC25 were transfected with a lentivirus-mediated ZEB1 overexpression, and Illumina microarrays analysis was performed. A total of 146 overlapping DEGs, including 74 upregulated and 72 downregulated genes, were identified from SCC9 and SCC25 cell lines. GO, and KEGG analysis revealed that these DEGs were primarily enriched in “cellular component organization or biogenesis,” “metabolic process,” “membrane-enclosed lumen,” “organelle part,” “extracellular region part,” and “membrane part.” Increasing evidence indicates that tumor-infiltrating immune cells could modulate tumor development. We also observed the association between the prognosis of ZEB1 and the infiltration of immune cells in OSCC. We found that the prognosis of ZEB1 was notably associated with tumor-infiltrating immune cells.

In conclusion, through microarrays analysis and bioinformatics analysis, the ZEB1 gene was identified as markedly associated with the OS of patients with OSCC. ZEB1 gene might serve as a novel prognostic marker that could be applied to forecast the prognosis of patients with OSCC. However, further examination of ZEB1 both in vivo and in vitro is needed to validate the results of the present study, prove the roles, and expose the potential mechanisms of OSCC.

The article "Comprehensive and Integrated Analysis Identifies ZEB1 as a Key Novel Gene in Oral Squamous Cell Carcinoma" was retracted in 2023. Reasons: signs of a paper mill; suspected computer-generated content; unreliable results or conclusions; concerns about the data.

## Figures and Tables

**Figure 1:** Differential expression of genes in the GSE58812 dataset from the GEO database. (a) A volcano plot of the GSE58812 data. DEGs were screened with |FC| > 2.0 and an adjusted *P* < 0.05. (b) The cluster heat map of the GSE58812 data.

**Figure 2:** Functional enrichment analysis. Upregulated DEGs (a) and downregulated DEGs (b) in GSE58812 data enriched in the GO pathway. (c) KEGG pathway enriched in GSE58812 data for common genes.

**Figure 3:** PPI network for common DEGs. PPI networks were constructed for the common DEGs.

**Figure 4:** Expression levels of ZEB1 in different tumors. The expression levels of ZEB1 in the integrated GTEx and TCGA dataset, total 33 tumors.

**Figure 5:** Univariate analysis of the prognostic value of ZEB1 expression in OSCC. (a) The expression level of ZEB1 is connected to clinicopathological traits of oral cancer. (b) ZEB1 was highly expressed in OSCC compared with normal tissues, and (c) was correlated with stage. (d) The cumulative survival rate of ZEB1 in OSCC. (e) Receiver operating characteristic analysis (ROC) of ZEB1 in OSCC. (f) The nomogram is applied by adding up the ZEB1 TPM value and stage plot, the total points projected on the bottom scales implied the probability of 1-, 3-, and 5-year survival.

**Figure 6:** Microarray analysis and screening of DEGs in OSCC. (a, b) DEGs were obtained for SCC9 and SCC25 cell lines, respectively. (c, d) Heatmap of common genes for SCC9 and SCC25 cell lines, respectively. (e, f) Venny map of differentially expressed genes among the two cell lines of DEGs, respectively.

**Figure 7:** Enrichment analysis of common genes. (a, b) The biological processes, cellular components, and molecular functions were enriched in common genes for the SCC9 and sSCC25 cell lines, respectively. (c, d) KEGG pathways enriched in common genes for the SCC9 and sSCC25 cell lines, respectively.

**Figure 8:** The association between the prognosis of ZEB1 and the infiltration of immune cells in OSCC. TIMER database was employed to examine the association between the prognosis of ZEB1 and the infiltration of immune cells in OSCC.

**Table 1:** Correlation of ZEB1 expression with clinicopathological features in the GSE30784 dataset.

Characteristic	Levels	ZEB1 expression		
		Low (%)	High (%)	
Age	≤60	53 (23.2%)	48 (21.1%)	0.107
	>60	61 (26.8%)	66 (28.9%)	

Gender	Female	59 (25.9%)	46 (20.1%)	0.230
	Male	55 (24.1%)	68 (29.8%)	

Clinical *T* category	*T*3-*T*4	52 (22.8%)	44 (19.3%)	**0.001**
	*T*1-*T*2	56 (24.6%)	60 (26.3%)	

Clinical *N* category	*N*+	61 (26.8%)	69 (30.3%)	0.068
	*N*0	9 (3.9%)	7 (3.1%)	

Pathologic stage	High	51 (22.4%)	54 (22.6%)	0.229
	Medium-low	63 (27.6%)	64 (27.4%)	

TNM staging	I-II	49 (20.5%)	53 (23.2%)	0.510
	III-IV	69 (29.5%)	61 (27.8%)	

Bold value implies *P* < 0.05.

The article "Comprehensive and Integrated Analysis Identifies ZEB1 as a Key Novel Gene in Oral Squamous Cell Carcinoma" was retracted in 2023. Reasons: signs of a paper mill; suspected computer-generated content; unreliable results or conclusions; concerns about the data.

**Table 2:** Screening DEGs in OSCC by microarray analysis.

DEGs	Gene terms
Upregulated	YTHDF2 CRYAB KLHDC10 C2CD2L VWDE CBLB TICAM2 NR4A2 CDC42EP5 FAM72A BSPRY ZC3H11A NKD2 CDK20 ZBTB43 ZNF791 C1QTNF12 RASA4 LIN52 ARMCX1 ISL1 SPACA4 TRMT44 INSIG2 FAM72C GSDMB ABCG1 ICAM3 CHKA C4A SEC13 CRIPT PPP1R32 ZNF568 ZNF674-AS1 LH X6 IT1 SNAI1 SNHG21 RNF150 NRTN ZNF256 YBX2 PNPLA8 KCTD20 ALDH6A1 SENP7 YOD1 TMEM59L P2RY11 LEPR RNASE4 CCDC186 UMAD1 KRTDAP TMED7 VCPKMT CDC37L1 EME2 MAP2 OVGP1 CST7 FAM83E PNLIPRP3 THAP2 RHPN1 B3GNT4 KLF7 RBAK ZEB1

Downregulated	LFNG FAM111B CALML3 KRT19 TAGLN SOCS1 ADM FGFBP1 MYBL2 APLN CSF2 ASF1B FHOD3 VIM RNASE7 CSF3 SFRP1 CXCL1 MCM5 FEZ1 CITED2 RRAD CAVIN3 RBBP8 ARVCF TECPR2 WDR76 IKBKE MSC ACKR3 SIRPA RASSF10 CSF1 TNFAIP3 HLA-V DPP3 HNRNPR SGK1 LRRC45 CHMP6 LPXN CSTF2 ZNF362 EID2 MFAP5 C1QTNF1 GINS3 TIMM8B RPL7L1 RBL1 CT62 CYGB CD83 EGLN3 DUBR PKIA
	PCDH7 P2RY2 DHFR LINP1 IVL ISM1 ZWINT MINDY4 RAB15 PKMYT1 CNTFR GDNF PLEC DHX9 STC1 DKK1 METTL16 E2F1

## Data Availability

The simulation experiment data used to support the findings of this study are available from the corresponding author upon request.
